The article "Gut Microbiota Is a Key Modulator of Insulin Resistance in TLR 2 Knockout Mice" was retracted in 2016. Reasons: errors in the images; duplicated images.

# Gut Microbiota Is a Key Modulator of Insulin Resistance in TLR 2 Knockout Mice

**DOI:** 10.1371/journal.pbio.1001212

**Published:** 2011-12-06

**Authors:** Andréa M. Caricilli, Paty K. Picardi, Lélia L. de Abreu, Mirian Ueno, Patrícia O. Prada, Eduardo R. Ropelle, Sandro Massao Hirabara, Ângela Castoldi, Pedro Vieira, Niels O. S. Camara, Rui Curi, José B. Carvalheira, Mário J. A. Saad

**Affiliations:** 1 Department of Internal Medicine, State University of Campinas, Campinas, Brazil; 2 Department of Nursing, State University of Campinas, Campinas, Brazil; 3 Department of Physiology and Biophysics, Institute of Biomedical Sciences, University of São Paulo, São Paulo, Brazil; 4 Department of Immunology, Institute of Biomedical Sciences, University of São Paulo, São Paulo, Brazil; University of Cambridge, United Kingdom

## Abstract

Environmental factors and host genetics interact to control the gut microbiota, which may have a role in the development of obesity and insulin resistance. TLR2-deficient mice, under germ-free conditions, are protected from diet-induced insulin resistance. It is possible that the presence of gut microbiota could reverse the phenotype of an animal, inducing insulin resistance in an animal genetically determined to have increased insulin sensitivity, such as the TLR2 KO mice. In the present study, we investigated the influence of gut microbiota on metabolic parameters, glucose tolerance, insulin sensitivity, and signaling of TLR2-deficient mice. We investigated the gut microbiota (by metagenomics), the metabolic characteristics, and insulin signaling in TLR2 knockout (KO) mice in a non-germ free facility. Results showed that the loss of TLR2 in conventionalized mice results in a phenotype reminiscent of metabolic syndrome, characterized by differences in the gut microbiota, with a 3-fold increase in Firmicutes and a slight increase in Bacteroidetes compared with controls. These changes in gut microbiota were accompanied by an increase in LPS absorption, subclinical inflammation, insulin resistance, glucose intolerance, and later, obesity. In addition, this sequence of events was reproduced in WT mice by microbiota transplantation and was also reversed by antibiotics. At the molecular level the mechanism was unique, with activation of TLR4 associated with ER stress and JNK activation, but no activation of the IKKβ-IκB-NFκB pathway. Our data also showed that in TLR2 KO mice there was a reduction in regulatory T cell in visceral fat, suggesting that this modulation may also contribute to the insulin resistance of these animals. Our results emphasize the role of microbiota in the complex network of molecular and cellular interactions that link genotype to phenotype and have potential implications for common human disorders involving obesity, diabetes, and even other immunological disorders.

The article "Gut Microbiota Is a Key Modulator of Insulin Resistance in TLR 2 Knockout Mice" was retracted in 2016. Reasons: errors in the images; duplicated images.

## Abstract 2

A genetic and pharmacological approach reveals novel insights into how changes in gut microbiota can subvert genetically predetermined phenotypes from lean to obese.

## Author Summary

An intricate interaction between genetic and environmental factors influences the development of obesity and diabetes. Previous studies have shown that mice lacking an important receptor of the innate immune system, Toll-like Receptor 2 (TLR2), are protected from insulin resistance. Given that the innate immune system has emerged as a key regulator of the gut microbiota, we undertook to investigate in this study whether the gut microbiota have a role in modulating the response to insulin. By rearing these TLR2 mutant mice in conventional facilities (as opposed to “germ-free” conditions) we figured that they would develop an altered gut microbiota. In contrast to previous studies, our results show that these TLR2 mutant mice now develop a diseased phenotype reminiscent of metabolic syndrome, including weight gain, and end up with gut microbiota similar to that found in obese mice and humans. These mice could be rescued by treatment with broad-spectrum antibiotics, which decimated the microbiota. Conversely, transplantation of the gut microbiota from these mice to wild-type mice induced weight gain and the metabolic syndrome phenotype. Our results indicate that the gut microbiota per se can subvert a genetically predetermined condition previously described as being protective towards obesity and insulin resistance into a phenotype associated with weight gain and its complications, such as glucose intolerance and diabetes.

## Introduction

The recent epidemics of obesity and type 2 diabetes mellitus (T2DM) in the past 20 years have stimulated researchers to investigate the mechanisms that are responsible for the development of these diseases. The general view is that obesity and T2DM have a genetic background and are strongly influenced by the environment and that insulin resistance is an early alteration in these diseases [1]–[5]. In addition, studies over the past 10 years have also shown that subclinical inflammation has an important role in the molecular mechanism of insulin resistance in obesity and T2DM [6]–[10]. During the past five years, an increasing body of literature has suggested other components of the mechanisms of these diseases that lie between the genetic and the environment factors, where the gut microbiota are now considered to make an important contribution to these mechanisms [11]–[16]. Then, it is now clear that environmental factors and host genetics interact to control the gut microbiota, which may have a role in the development of obesity and insulin resistance [17].

The article "Gut Microbiota Is a Key Modulator of Insulin Resistance in TLR 2 Knockout Mice" was retracted in 2016. Reasons: errors in the images; duplicated images.

Metagenomic studies demonstrated that the proportion of Firmicutes is higher in obese animals and in humans, compared with lean controls, and this correlates with a higher number of genes encoding enzymes that break down otherwise indigestible dietary polysaccharides, with more fermentation end products and fewer calories remaining in the faeces of obese individuals [18],[19]. Another mechanism by which the microbiome may contribute to metabolic disorders is by triggering systemic inflammation [20]. The immune system coevolves with the microbiota during postnatal life, which allows the host and microbiota to coexist in a mutually beneficial relationship [21],[22]. In particular, the innate immune system has emerged as a key regulator of the gut microbiota. Innate immune recognition of microbe-associated molecular patterns is executed by families of pattern-recognition molecules with a special role for Toll-like receptors (TLRs) [23],[24]. Recent findings indicate that TLRs, which are up-regulated in the affected tissue of most inflammatory disorders, can mediate crosstalk between the immune systems and whole body metabolism [23]. It has been demonstrated that TLR4, a sensor for lipopolysaccharides on Gram-negative bacteria, is involved in the induction of proinflammatory cytokine expression in macrophages, adipocytes, and liver [13],[25]. We and others have demonstrated that TLR4 genetically deficient mice or mice with an inactivating mutation for this receptor are substantially protected from obesity-induced insulin resistance [26],[27]. Similarly, TLR2 genetically deficient mice are protected from high-fat-induced insulin resistance [28],[29]. On the other hand, TLR5-deficient mice exhibit hyperphagia and develop hallmark features of metabolic syndrome, including hyperlipidemia, hypertension, insulin resistance, and increased adiposity [30], and these alterations are the consequence of alterations in the gut microbiota. It is important to emphasize that the studies that investigated TLR4- and TLR5-deficient mice were performed without germ-free conditions [26],[27],[30], suggesting that the microbiota have an important influence on TLR5-deficient mice phenotype, inducing obesity and insulin resistance; however, in the TLR4-deficient mice, the microbiota do not have a role in these phenomena because these animals are protected from diet-induced insulin resistance, independently of germ-free conditions [26],[27]. Taken together, these findings suggest that the interaction of the innate immune system with gut microbiota may determine the insulin sensitivity of an animal and that TLRs may have different roles in this process. Since in most studies with TLR2-deficient mice the microbiota were not investigated, we cannot predict the influence of microbiota in the protection or in the development of insulin resistance in these mice. It is possible that the presence of a diverse gut microbiota could completely reverse the phenotype of an animal, inducing insulin resistance in an animal genetically determined to have increased insulin sensitivity, such as the TLR2 KO mice. The aim of the present study was to investigate the influence of gut microbiota in metabolic parameters, glucose tolerance, insulin sensitivity, and signaling of TLR2-deficient mice.

The article "Gut Microbiota Is a Key Modulator of Insulin Resistance in TLR 2 Knockout Mice" was retracted in 2016. Reasons: errors in the images; duplicated images.

## Results

### Animal Characteristics

TLR2 KO mice did not present any difference in weight gain, compared with their controls up until 12 wk. However, after 12 wk, TLR2 KO mice were heavier than their controls (*p*<0.05; Figure 1A). No significant differences were observed with regard to food intake between the groups after either 8 or 16 wk (Figure 1B). The food intake was also normalized for body weight and no difference was observed between groups at 8 wk old (WT = 0.22±0.035 g/g animal/day; TLR2 KO = 0.21±0.021 g/g animal/day). However, after 16 wk, TLR2 KO mice presented increased epididymal fat weight (Figure 1C). After 12 wk, the amount of adipose tissue is visually increased in TLR2 KO mice (Figure 1D). It is interesting that TLR2 KO mice at 8 wk old had decreased glucose tolerance compared to their controls (*p*<0.05; Figure 1E), but no difference was observed in fasting serum insulin between the groups (Figure 1F). We next submitted these animals to a hyperinsulinemic euglycemic clamp to investigate insulin sensitivity; results showed that TLR2 KO mice presented a significant decrease in the rate of glucose uptake under high insulin stimulus (50% of control, *p*<0.05; Figure 1G), indicating a clear situation of insulin resistance.

**Figure 1:** Metabolic parameters of TLR2 knockout (TLR2^−/−^) and WT mice during 16 wk. (A) Weight gain after 16 wk. (B) Food intake after 8 and 16 wk. (C) Epididymal fat pad weight after 8 and 16 wk. (D) WT and TLR2−/− mice after 20 wk. (E) Glucose tolerance test. (F) Serum insulin concentration. (G) Glucose uptake obtained from euglycaemic hyperinsunaemic clamp. (H) Oxygen consumption and (I) respiratory exchange rate. (J) UCP-1 expression in the brown adipose tissue. Equal protein loading in the gel was confirmed by reblotting the membrane with an anti-β-actin antibody (J, lower panel). All evaluations were made with mice on standard chow. Data are presented as means ± S.E.M from six to eight mice per group from experiments that were repeated at least three times. *p<0.05 between TLR2−/− mice and their controls.

The article "Gut Microbiota Is a Key Modulator of Insulin Resistance in TLR 2 Knockout Mice" was retracted in 2016. Reasons: errors in the images; duplicated images.

We next analyzed the oxygen consumption from both groups and observed that TLR2 KO mice presented decreased oxygen consumption (Figure 1H), suggesting decreased energy expenditure when compared with their controls. However, the respiratory exchange ratio, approximately 0.85, was similar between the groups (Figure 1I). As the oxygen consumption was decreased in TLR2 KO mice, we evaluated a marker of thermogenesis in the brown adipose tissue of both groups. The expression of the thermogenesis-inducing protein, UCP1, was significantly decreased in TLR2 KO mice (Figure 1J), suggesting reduced energy expenditure in these animals, in accordance with the reduced oxygen consumption observed.

In order to characterize the gut microbiota of TLR2 KO mice, we pyrosequenced the 16S ribosomal RNA (rRNA) from the stools of these animals. TLR2 KO mice presented a different gut microbiota, compared with their controls. The major difference concerns the proportion of Firmicutes, which was approximately 47.92% in TLR2 KO mice, while the controls presented a proportion of 13.95%. Moreover, TLR2 KO mice presented 47.92% Bacteroidetes and 1.04% Proteobacteria, while their controls presented approximately 42.63% and 39.53%, respectively (Figure 2A,B). TLR2 KO mice presented other differences in regards to classes and families and these results are presented in the Supporting Information section (Figures S1 and S2).

**Figure 2:** TLR2 KO mice exhibit taxonomical alterations in gut microbiota. Untreated WT (A) and TLR2 knockout (TLR2−/−) mice (B) stools were analyzed via 16S rRNA analysis. Data are presented from six to eight mice per group from experiments that were repeated at least three times. All evaluations were made with mice on standard chow.

However, it is important to notice that we have observed different proportions of these phyla between TLR2 KO mice and their controls in different ages of mice. From 4-wk-old to 1-y-old mice, we observed increased proportion of Firmicutes in TLR2 KO mice compared with the controls. We have also observed a tendency of decreasing the proportion of Bacteroidetes progressively as TLR2 KO mice get older (Figures S3, S4, S5).

### Molecular Mechanisms of Insulin Resistance in TLR2 KO Mice

Next, we determined the serum concentration of IL-6 and TNF-α in both groups of animals and observed that TLR2 KO mice presented reduced levels of these cytokines compared with their controls (Figure 3A,B). We also investigated the serum concentrations of leptin, adiponectin, and LPS. No significant difference was observed between the groups with regard to leptin and adiponectin (Figure 3C,D). On the other hand, LPS serum concentration was increased in TLR2 KO mice (Figure 3E).

The article "Gut Microbiota Is a Key Modulator of Insulin Resistance in TLR 2 Knockout Mice" was retracted in 2016. Reasons: errors in the images; duplicated images.

**Figure 3:** Measurements of cytokines, adipokines, and LPS. Serum concentration of IL-6 (A), TNF-α (B), adiponectin (C), leptin (D), and LPS (E). Proportion of *Bifidobacterium* was obtained by 16S rRNA analysis of stools (F). Data are presented as means ± S.E.M from six to eight mice per group from experiments that were repeated at least three times. * *p*<0.05 between TLR2 KO mice and their controls; all evaluations were made with mice on standard chow.

As TLR2 KO mice presented increased serum LPS levels, and this alteration was previously described in an animal model of obesity in which there was a reduced proportion of *Bifidobacterium* [31], we investigated the proportion of this group of bacteria. We observed that TLR2 KO mice presented a decrease in *Bifidobacterium* proportion compared with WT (Figure 3F).

In order to unravel the mechanism by which the insulin resistance occurs in the TLR2 KO mice, we studied important pathways involved in this phenomenon: phosphorylation of JNK, activation of ER stress, serine phosphorylation of the insulin receptor substrate (IRS)-1, and expression of IκB-α, which is involved in the inhibition of the IKK/NFκB pathway activation.

TLR2 KO mice presented increased phosphorylation of JNK in muscle, liver, and adipose tissue compared with controls (Figure 4A–C). Since the activation of ER stress leads to the phosphorylation of JNK, the increased phosphorylation of this protein in TLR2 KO mice could be due to this event. In fact, the phosphorylation of PERK was increased in the liver and adipose tissue of the KO mice, suggesting increased ER stress activation at least in these two tissues (Figure 4D–F).

**Figure 4:** Evaluation of pathways involved in the impairment of insulin signaling. Phosphorylation of JNK in muscle (A), liver (B), and white adipose tissue (WAT) (C). Phosphorylation of PERK in muscle (D), liver (E), and WAT (F). Serine 307 phosphorylation of IRS-1 from muscle (G), liver (H), and WAT (I). Activation of TLR4 (studied by the immunoprecipitation of MyD88 and blotting with TLR4) in muscle (J), liver (K), and WAT (L). JNK, PERK, and IRS-1 protein expression in muscle, liver, and white adipose tissue (A–I, lower panels). Expression of IκB-α in muscle (M), liver (N), and WAT (O). Equal protein loading in the gel was confirmed by reblotting the membrane with an anti-β-actin antibody (M–O, lower panels). NFκB activation in muscle (P), liver (Q), and WAT (R). All evaluations were made with mice on standard chow. Data are presented as means ± S.E.M from six to eight mice per group from experiments that were repeated at least three times. * *p*<0.05 between TLR2−/− mice and their controls.

The article "Gut Microbiota Is a Key Modulator of Insulin Resistance in TLR 2 Knockout Mice" was retracted in 2016. Reasons: errors in the images; duplicated images.

Next, we studied the inhibitory serine phosphorylation of IRS-1 in muscle, liver, and adipose tissue of TLR2 KO mice and observed that this phosphorylation was increased, compared with the controls, suggesting impairment of insulin signaling (Figure 4G–I). Since increased serum concentration of LPS, a TLR4 ligand, was observed in TLR2 KO mice, we investigated the activation of TLR4 in the muscle, liver, and adipose tissue of these mice. An increased activation of this receptor was observed in all tissues studied (Figure 4J–L), suggesting that, in the absence of TLR2, a compensatory action may lead to increased activation of TLR4, which may also contribute to the development of insulin resistance in TLR2 KO mice.

Then, we studied the activation of IKK/NFκB pathway, indirectly, by the expression of IκB-α. Curiously, the expression of IκB-α was increased in the muscle, liver, and white adipose tissue of TLR2 KO mice, compared with controls, suggesting a decreased activation of IKK/NFκB pathway (Figure 4M–O). In order to confirm this result, we studied the activation of NFκB and observed that this was decreased in all tissues studied from TLR2 KO mice (Figure 4P–R).

The insulin-induced tyrosine phosphorylation of the insulin receptor (IR) (Figure S6A–C) and of the insulin receptor substrate (IRS)-1 (Figure 5A–C), as well as the insulin-induced serine phosphorylation of AKT, was decreased in the muscle, liver, and adipose tissue of TLR2 KO mice (Figure 5D–F), compared with their controls, suggesting reduced insulin signaling in these tissues.

**Figure 5:** TLR2 knockout (TLR2−/−) mice present decreased insulin signaling. Tyrosine 941 phosphorylation of the insulin receptor substrate (IRS)-1 in muscle (A), liver (B), and WAT (C). Serine phosphorylation of AKT in muscle (D), liver (E), and WAT (F). IRS-1 and AKT protein expression in muscle, liver, and white adipose tissue (A–F, lower panels). Equal protein loading in the gel was confirmed by reblotting the membrane with an anti-β-actin antibody (lower panels). All evaluations were made with mice on standard chow. Data are presented as means ± S.E.M from six to eight mice per group from experiments that were repeated at least three times. *p<0.05 between WT with and without insulin stimulus; ** *p*<0.05 between TLR2−/− mice and their controls with insulin stimulus.

Other proteins that are important in the modulation of insulin action were also investigated. Our data showed that the phosphorylation of AMPK (Figure S6D–F) and the expression of PGC-1α (Figure S6G–I) were similar between controls and TLR2 KO mice in the three tissues investigated.

The article "Gut Microbiota Is a Key Modulator of Insulin Resistance in TLR 2 Knockout Mice" was retracted in 2016. Reasons: errors in the images; duplicated images.

As an increased phosphorylation of JNK was observed in TLR2 KO mice, we prevented the activation of this protein with a pharmacological inhibitor, SP600125, by treating mice with daily i.p. injections for 5 d. Subsequently, we observed an increased glucose uptake in these animals, suggesting that the activation of JNK is indeed relevant to the development of insulin resistance (Figure 6A). We also observed increased insulin-induced serine phosphorylation of AKT in the liver (Figure 6B), muscle, and white adipose tissue (unpublished data) of TLR2 KO mice after this treatment, suggesting increased insulin signaling, as well, associated with a reduction in JNK phosphorylation in the liver of TLR2 KO mice (Figure 6D).

**Figure 6:** Insulin sensitivity and signaling after treatment with selective inhibitors. Glucose uptake obtained by the euglycaemic hyperinsulinaemic clamp from TLR2−/− mice treated or not with the drugs: SP600125 (SP), JNK inhibitor; 4-phenil butyric acid (PBA), endoplasmic reticulum stress inhibitor; TLR4 antisense oligonucleotide (ASO); (A) TAK-242, inhibitor of TLR4. (B) Serine phosphorylation of AKT after the treatment with SP600125 and PBA. (C) Serine phosphorylation of AKT after the treatment with TLR4 ASO and TAK-242. (D) Phosphorylation of JNK after the treatment with the drugs mentioned. Fasted TLR2 knockout mice and WT mice were gavaged by LPS (1.08, 10^−8^ g) diluted in water (100 µL) or without LPS. (E) Blood was collected from the cava vein 60 min after gavage and serum LPS was determined. (F) Zonula occludens (ZO)-1 expression in the ileum. (G) Frequency of CD4+Foxp3+ regulatory T cells in WT mice. (H) Frequency of CD4+Foxp3+ regulatory T cells in TLR2−/− mice. All evaluations were made with mice on standard chow. Data are presented as means ± S.E.M from six to eight mice per group from experiments that were repeated at least three times. * *p*<0.05 between WT mice with or without insulin stimulus; ** *p*<0.05 between WT and TLR2−/− mice with insulin stimulus ; $ *p*<0.05 between TLR2−/− mice with insulin stimulus, treated or not with SP; # *p*<0.05 between TLR2−/− mice with insulin stimulus, treated or not with PBA; § *p*<0.05 between TLR2−/− mice with insulin stimulus, treated or not with ASO; & *p*<0.05 between TLR2−/− mice with insulin stimulus, treated or not with TAK-242; ^a^ *p*<0.05 between WT mice with or without LPS stimulus; ° *p*<0.05 between WT and TLR2−/− mice with LPS stimulus.

An increased activation of ER stress leads to the activation of JNK [32],[33]. Therefore, we studied whether preventing the activation of this phenomenon could improve the insulin sensitivity and signaling. For this purpose, we treated mice with a pharmacological inhibitor of ER stress, 4-phenyl butyric acid (PBA), using i.p. daily injections for 10 d. This treatment was found to lead to an increased glucose uptake in TLR2 KO mice (Figure 6A) and increased insulin-induced serine phosphorylation of AKT in the liver (Figure 6B), muscle, and white adipose tissue (unpublished data), suggesting an improvement in the insulin signaling as well. After this treatment, we also investigated the phosphorylation of JNK and observed a reduction in the liver (Figure 6D) of TLR2 KO mice. Results suggest that both the activation of ER stress and the activation of JNK are important contributors to the development of the phenotype observed in TLR2 KO mice.

The article "Gut Microbiota Is a Key Modulator of Insulin Resistance in TLR 2 Knockout Mice" was retracted in 2016. Reasons: errors in the images; duplicated images.

Since TLR4 was more activated in the tissues of TLR2 KO mice, possibly constituting one of the mechanisms responsible for the development of insulin resistance, we inhibited its expression using a TLR4 antisense oligonucleotide (ASO; with two daily i.p. injections) for 5 d. After TLR4 ASO treatment, TLR2 KO mice were found to present a significantly increased glucose uptake during the euglycemic hyperinsulinemic clamp compared with their controls (Figure 6A). The insulin signaling was also increased, with increased insulin-induced serine phosphorylation of AKT in the liver (Figure 6C), muscle, and white adipose tissue (unpublished data) of TLR2 KO mice. After this treatment, decreased phosphorylation of JNK was observed in the liver (Figure 6D) of TLR2 KO mice.

Using another method to inhibit TLR4 signaling, a pharmacological inhibitor of TLR4, TAK-242, was administered daily by gavage during 5 d and confirmed the results seen with the TLR4 ASO treatment. The insulin sensitivity was increased in TLR2 KO-treated animals (Figure 6A), and the insulin-induced serine phosphorylation of AKT was also increased in the liver (Figure 6C) of these animals, suggesting an improvement in insulin signaling. The phosphorylation of JNK was decreased in the liver (Figure 6D) of TLR2 KO treated mice.

As the serum LPS levels were increased in TLR2 KO mice, and the changes in microbiota may not account for this increase, we tested whether the LPS absorption was also increased in these animals. For this purpose, we administered LPS orally to TLR2 KO mice and wild type mice and determined the circulating LPS levels 1 h later. We observed that all animals presented increased serum LPS concentration after the LPS administration. However, TLR2 KO mice presented a higher increase in serum LPS concentration after the treatment, compared with the wild type mice (Figure 6E). As this result suggested that TLR2 KO mice presented increased gut permeability, we investigated the expression of an important tight-junction protein of the ileum of these mice, zonula occludens (ZO)-1, and observed that it was indeed decreased, compared with the control mice (Figure 6F). Reduction of ZO-1 expression in TLR2 KO mice was also observed in other parts of the small intestine and in the colon (unpublished data).

The article "Gut Microbiota Is a Key Modulator of Insulin Resistance in TLR 2 Knockout Mice" was retracted in 2016. Reasons: errors in the images; duplicated images.

Previous data showed that TLR2 KO mice have a decreased number of regulatory T cells in the circulation compared with control mice [34]. This can have a role in the modulation of intestinal barrier and also in insulin resistance. We next investigated the frequency of Foxp3+ CD4+ T regulatory cells in mesenteric adipose tissue. We observed that the frequency of these cells was decreased in TLR2 KO mice (Figure 6H), compared with the wild type mice (Figure 6G).

### Treatment of TLR2 KO Mice with Antibiotics Changes the Composition of Their Gut Microbiota and Improves Insulin Sensitivity

As the gut microbiota from TLR2 KO mice was shown to differ from that of controls, we treated both groups with a mixture of antibiotics (ampicillin, neomycin, and metronidazole) in their drinking water for 20 d. Moreover, we characterized the gut microbiota of TLR2 KO mice using culture-based microbial analysis of cecal contents after the antibiotics treatment and the results showed that aerobic bacteria were almost suppressed, while anaerobic bacteria decreased its abundance to 40% compared to the control group (Figure S7A).

After the treatment with the mixture of antibiotics, we also observed changes in the relative abundance of three phyla of bacteria. The abundance of Bacteroidetes was reduced from 47.92% to 19.78% and Firmicutes abundance decreased from 47.92% to 11.76% in the TLR2 KO mice, while Proteobacteria abundance increased from 1.04% to 67.38% in these mice (Figure S7B,C). TLR2 KO treated mice presented other differences in regards to classes and families and these results are presented in the Supporting Information section (Figures S8 and S9). When TLR2 KO mice were treated with metronidazole, neomycin, and ampicillin individually, and not as an antibiotics mixture, we observed that ampicillin was the most effective one to exterminate more bacteria diversity. When treated with metronidazole, TLR2 KO mice presented 46.51% of Proteobacteria, 10.69% of Firmicutes, and 42.32% of Bacteroidetes. When treated with neomycin, TLR2 KO mice presented 44.18% of Firmicutes and 55.81% of Bacteroidetes. When treated with ampicillin, almost 100% of the sequenced bacteria left corresponded to Proteobacteria (Figure S10A–C). Since the treatment with ampicillin or metronidazole normalized glucose tolerance in TLR2 KO mice, and neomycin only mildly improved glucose tolerance in these mice (unpublished data), we can speculate that the changes in microbiota induced by ampicillin or metronidazole are more relevant than the changes induced by neomycin, although no specific genera of bacteria can be implicated in this response. However, in accordance with previous data on obese mice, the decrease in the proportion of the phylum Firmicutes, as observed in the groups that received ampicillin or metronidazole, correlates with the improvement in glucose tolerance.

The article "Gut Microbiota Is a Key Modulator of Insulin Resistance in TLR 2 Knockout Mice" was retracted in 2016. Reasons: errors in the images; duplicated images.

TLR2 KO mice presented decreased epididymal fat pad and visceral adipose tissue weight after the treatment with antibiotics compared with non-treated TLR2 KO, while no difference was observed in the treated and non-treated control animals (Figure 7A,B). TLR2 KO mice also presented increased glucose tolerance (Figure 7C) and increased oxygen consumption (Figure 7D) after the treatment compared with non-treated TLR2 KO mice, but no significant difference was observed between treated and non-treated control mice. With regard to insulin sensitivity and signaling, we observed an improvement in insulin-induced glucose uptake, using the euglycemic hyperinsulinemic clamp, in TLR2 KO mice after antibiotics treatment (Figure 7E), with no difference in the treated and non-treated control mice. After the treatment, we also observed an increase in the UCP-1 expression in the brown adipose tissue of TLR2 KO mice, supporting the increased oxygen consumption observed in this condition (Figure 7F). We also observed an increased insulin-induced serine phosphorylation of AKT in the liver (Figure 7G), muscle, and white adipose tissue (unpublished data) of TLR2 KO mice after the treatment. Moreover, there was a decreased phosphorylation of JNK in the liver (Figure 7H), muscle, and white adipose tissue (unpublished data) of the knockout mice after the treatment. The antibiotics treatment also led to an increased expression of ZO-1 in TLR2 KO mice, with no difference in the treated and non-treated control mice (Figure 7I). These data suggest that, in TLR2 KO mice, the reduction in their gut microbiota associated with qualitative changes in composition, induced by antibiotics, was able to reverse the insulin resistance of these animals.

**Figure 7:** Alterations in the metabolic parameters and in insulin signaling and sensitivity after treatment with antibiotics. (A) Epididymal fat pad weight. (B) Visceral adipose tissue weight. (C) Glucose tolerance test. (D) Oxygen consumption. (E) Glucose uptake obtained by the euglycaemic hyperinsulinaemic clamp. (F) UCP-1 expression in the brown adipose tissue. (G) Serine phosphorylation of AKT after the treatment with AB. (H) Phosphorylation of JNK after the treatment with AB. (I) Zonula occludens (ZO)-1 expression in the ileum. Equal protein loading in the gel was confirmed by reblotting the membrane with an anti-β-actin antibody (lower panels). Data are presented as means ± S.E.M from six to eight mice per group, from experiments that were repeated at least three times. All evaluations were made with mice on standard chow. # *p*<0.05 between WT mice with or without insulin stimulus; * *p*<0.05 between WT and TLR2−/− mice with insulin stimulus; ** *p*<0.05 between TLR2−/− and TLR2−/− treated with AB, with insulin stimulus.

The article "Gut Microbiota Is a Key Modulator of Insulin Resistance in TLR 2 Knockout Mice" was retracted in 2016. Reasons: errors in the images; duplicated images.

### Effect of Microbiota Transplantation from TLR2 KO Mice to Control Mice on Weight Gain and Insulin Sensitivity

In order to investigate whether the gut microbiota was responsible for triggering all the alterations seen in TLR2 KO mice, we transplanted the cecal microbiota from TKR2 KO mice and from WT mice in 4-wk-old-*Bacillus*-associated WT mice, which contain few species of the genus *Bacillus*, without any other genera, as obtained by 16S rRNA pyrosequencing, in the following proportion: *Bacillus simplex* (0.68%), *Bacillus sp* (1.1%), *Bacillus sp* Kaza-34 (6.28%), and uncultured *Bacillus* (91.96%). There was a non-significant increase in the epididymal adipose tissue fat pad weight, in the total body weight gain, in the fasting blood glucose, and in the oxygen consumption in *Bacillus*-associated mice transplanted with WT microbiota (Figure 8A,C,D,G). However, in *Bacillus*-associated mice transplanted with TLR2 KO microbiota, we observed a marked increase in the epididymal fat pad and visceral adipose tissue weight (Figure 8A,B); in the body weight gain (Figure 8C), with a trend towards increased fasting blood glucose (Figure 8D), as well as a decrease in the glucose tolerance (Figure 8E,F); in the oxygen consumption (Figure 8G); and in the insulin sensitivity, obtained by euglycemic hyperinsulinemic clamp, compared with those transplanted with WT microbiota (Figure 8H) 8 wk after the transplantation (*p*<0.05). *Bacillus*-associated mice transplanted with WT microbiota also presented decreased insulin sensitivity compared with the non-transplanted mice (*p*<0.05). *Bacillus*-associated WT mice transplanted with TLR2 KO or with WT microbiota also showed decreased expression of UCP-1 in the brown adipose tissue compared with the non-transplanted mice. *Bacillus*-associated mice transplanted with TLR2 KO microbiota showed marked decrease in UCP-1 expression compared with those transplanted with WT microbiota (Figure 8I). Moreover, these animals had decreased insulin signaling, as seen by the reduction in serine phosphorylation of AKT in liver, compared to mice transplanted with WT microbiota (Figure 8J). In the mice transplanted with TLR2 KO microbiota, there was increased phosphorylation of JNK in liver (Figure 8K), muscle, and white adipose tissue (unpublished data) compared with the mice transplanted with WT microbiota. The experiments described above had also been performed in few germ-free mice, but with very similar results (unpublished data).

The article "Gut Microbiota Is a Key Modulator of Insulin Resistance in TLR 2 Knockout Mice" was retracted in 2016. Reasons: errors in the images; duplicated images.

**Figure 8:** WT mice reproduce TLR2 knockout (TLR2−/−) mice after cecal microbiota transplantation. (A) Epididymal fat pad weight. (B) Visceral adipose tissue weight. (C) Weight gain of transplanted mice. (D) Serum glucose. (E) Glucose tolerance test. (F) Incremental area under curva (IAUC) obtained from the glucose tolerance test. (G) Oxygen consumption. (H) Glucose uptake obtained by the euglycaemic hyperinsulinaemic clamp. (I) UCP-1 expression in the brown adipose tissue. (J) Serine phosphorylation of AKT after the treatment with AB. (K) Phosphorylation of JNK after the treatment with AB. AKT and JNK protein expression in the liver of transplanted mice (J, K, lower panels). (L) Zonula occludens (ZO)-1 expression in the ileum. (M) Frequency of CD4+Foxp3+ regulatory T cells in *Bacillus*-associated mice. (N) Frequency of CD4+Foxp3+ regulatory T cells in *Bacillus*-associated mice transplanted with WT microbiota. (O) Frequency of CD4+Foxp3+ regulatory T cells in *Bacillus*-associated mice transplanted with TLR2−/− microbiota. Equal protein loading in the gel was confirmed by reblotting the membrane with an anti-β-actin antibody (lower panels). Data are presented as means ± S.E.M from six to eight mice per group from experiments that were repeated at least three times. All evaluations were made with mice on standard chow. * *p*<0.05 between *Bacillus*-associated mice transplanted with TLR2−/− microbiota (MA+TLR2−/−) and those transplanted with WT microbiota (MA+WT); ** *p*<0.05 between *Bacillus*-associated mice transplanted with WT microbiota (MA+WT) and *Bacillus*-associated mice (MA); # *p*<0.05 between *Bacillus*-associated mice with or without insulin stimulus.

Eight weeks after the transplantation, the expression of ZO-1 was evaluated in the 12-wk-old mice. We observed that it was decreased in mice transplanted with TLR2 KO microbiota compared to those transplanted with WT microbiota (Figure 8L). The same data were observed in other parts of the small intestine and in the colon (unpublished data).

We also investigated the frequency of CD4+Foxp3+ regulatory T cells in these animals and observed that they were decreased in mesenteric adipose tissue in mice transplanted with TLR2 KO microbiota (Figure 8O) compared with the mice transplanted with WT microbiota (Figure 8N) and non-transplanted *Bacillus*-associated mice (Figure 8M).

The article "Gut Microbiota Is a Key Modulator of Insulin Resistance in TLR 2 Knockout Mice" was retracted in 2016. Reasons: errors in the images; duplicated images.

In summary, as expected, the transplantation of a wild-type microbiota in *Bacillus*-associated mice resulted in a moderate increase in adipose visceral fat and in a mild decrease in glucose tolerance. However, the effect of the transplantation of TLR2 KO microbiota in *Bacillus*-associated mice induced marked changes, and clearly indicates deleterious effects of this TLR2 KO microbiota on body weight and glucose metabolism.

### Effect of High-Fat Diet (HFD) on Weight Gain and Insulin Sensitivity in TLR2 KO Mice

Next, we investigated the effect of high-fat diet (HFD) on metabolic parameters of TLR2 KO mice. The results showed that at 8 wk old TLR2 KO mice on a HFD presented increased body weight (Figure 9A), similar food intake (WT = 7.3 g per day, TLR2 KO = 6.1 g per day; WT = 0.25±0.055 g/g animal/day; TLR2 KO = 0.19±0.046 g/g animal/day) (Figure 9B), increased epididymal fat weight (Figure 9C), reduced glucose tolerance (Figure 9D), increased fasting serum insulin (Figure 9E), and reduced glucose uptake (Figure 9F) compared to the controls. The oxygen consumption of both groups was compared and TLR2 KO mice were seen to present decreased oxygen consumption (Figure 9G), suggesting decreased energy expenditure compared to the controls. However, the respiratory exchange ratio was similar in both groups, being around 0.75 (Figure 9H). In accordance with the reduced oxygen consumption observed, the expression of UCP1 was significantly decreased in TLR2 KO mice (Figure 9I). Similarly, insulin signaling was reduced in TLR2 KO mice fed on the HFD. The insulin-induced serine phosphorylation of AKT was reduced in the muscle, liver, and white adipose tissue of TLR2 KO mice, compared with controls (Figure 10A–C). Moreover, the phosphorylation of JNK was increased in all tissues studied of the TLR2 KO mice (Figure 10D–F), while the expression of IκB-α was increased (Figure 10G–I), suggesting that the IKK/NFκB pathway is decreased in TLR2 KO mice on a HFD, as observed for mice on a standard chow. These results suggest that the metabolic phenotype of the TLR2 KO mice characterized by insulin resistance is aggravated by HFD, which leads to the development of diabetes, as demonstrated by fasting blood glucose and glucose tolerance tests.

**Figure 9:** Metabolic parameters of TLR2 KO (TLR2−/−) mice fed a high-fat diet. (A) Weight gain after 10 wk of high-fat diet (HFD). (B) Food intake. (C) Epididymal fat pad weight. (D) Glucose tolerance test. (E) Serum insulin concentration. (F) Glucose uptake obtained from the euglycaemic hyperinsulinaemic clamp. (G) Oxygen consumption and (H) respiratory exchange rate. (I) UCP-1 expression in the brown adipose tissue. Data are presented as means ± S.E.M from six to eight mice per group from experiments that were repeated at least three times. All evaluations were made with mice on standard chow. * *p*<0.05 between TLR2−/− mice and their controls.

The article "Gut Microbiota Is a Key Modulator of Insulin Resistance in TLR 2 Knockout Mice" was retracted in 2016. Reasons: errors in the images; duplicated images.

**Figure 10:** Insulin signaling is impaired in TLR2 knockout (TLR2−/−) mice fed on a high-fat diet. Phosphorylation of AKT in muscle (A), liver (B), and white adipose tissue (WAT) (C). AKT protein expression in muscle, liver, and WAT (A–C, lower panels). Phosphorylation of JNK in muscle (D), liver (E), and WAT (F). JNK protein expression in muscle, liver, and WAT (D–F, lower panels). IκB-α expression in muscle (G), liver (H), and WAT (I). Equal protein loading in the gel was confirmed by reblotting the membrane with an anti-β-actin antibody (lower panels). All evaluations were made with mice on standard chow. Data are presented as means ± S.E.M from six to eight mice per group from experiments that were repeated at least three times. * *p*<0.05 between TLR2−/− mice and their controls, with insulin stimulus; ** *p*<0.05 between WT with and without insulin stimulus.

## Discussion

It is now considered that environmental factors and host genetics interact to control the acquisition and stability of gut microbiota. In turn, environment, host genetics, and microbiota interact to maintain the homeostasis of gut, weight control, and insulin sensitivity [17]. Clearly, the modification of one or more of these three components may trigger the development of insulin resistance and obesity. The results of the present study demonstrated that TLR2 KO mice in conventionalized conditions in our breeding center have insulin resistance and glucose intolerance associated with alterations in the composition of the gut microbiota, which displayed an increase in the relative abundance of Firmicutes and Bacteroidetes and decreased relative abundance of Proteobacteria, compared to their controls. The insulin resistance of TLR2 KO mice was accompanied by a down-modulation of insulin-induced insulin signaling in the liver, muscle, and adipose tissue, associated with an increase in endoplasmic reticulum stress. These metabolic alterations were characterized in 8-wk-old TLR2 KO mice, when they had similar body weights to the control animals. As demonstrated in other animal models [35],[36], this insulin resistance precedes the development of obesity, and an augmentation in body weight compared to controls is observed after the 12th wk of age.

The article "Gut Microbiota Is a Key Modulator of Insulin Resistance in TLR 2 Knockout Mice" was retracted in 2016. Reasons: errors in the images; duplicated images.

However, previous studies [28],[37] have reported that TLR2 KO mice present decreased body weight and adiposity, are protected against insulin resistance, and gain less weight on a HFD than control mice and are also protected against related comorbidities [38],[39]. We believe that the main difference between these studies and our study may be related to gut microbiota. It should be taken into consideration that although the animals have the same genetic deficiency they were bred in different rooms and fed with food from different sources, which can certainly have a role in the establishment and maintenance of gut microbiota. Although in most of the previous studies the gut microbiota was not investigated, we can suggest that TLR2 deficiency associated with different environmental conditions can induce different phenotypes, probably induced by different microbiotas. Kellermayer et al. have shown that the proportion of Firmicutes found in TLR2 KO mice was lower than in WT, while the proportion of Bacteroidetes was increased [40]. In our study, we show that TLR2 KO mice present the opposite, with increased proportion of Firmicutes and decreased proportion of Bacteroidetes, compared with the WT. This way, it is possible that in the other published studies the proportions of this phyla might be different, compared with the proportions we have found, which might influence differently the phenotype observed. These results reinforce the importance of environment and of the innate immune system as key regulators of gut microbiota and suggest that a genetic condition, which by itself can prevent insulin resistance in some conditions, can also overcome the protective effect on insulin resistance in other environmental conditions inducing more weight gain, probably due to differences in the microbiota. In addition, these findings may help explain differences in the metabolic behavior of the same animal, when analyzed in distinct environments, and can contribute to explaining differences in metabolic behavior between animals with the same background or with the same genetic alteration.

The mechanisms by which the TLR2 KO mice presented insulin resistance and, later, obesity were also investigated. The gut microbiota of the TLR2 KO animal have some similarities to those found in obese animals and humans, with an increase in Firmicutes [41],[42]. This type of microbiota is usually associated with an increased capacity for energy harvesting from the diet [19]. This might contribute to explaining the obesity observed, but does not explain why these animals are clearly insulin resistant many weeks before they start to gain more weight than their controls. In addition, it was demonstrated that germ-free (that gain less weight on HFD) and conventionalized mice have similar energy contents in their feces, suggesting that other mechanisms may have an important role in gut microbiota-induced insulin resistance and obesity [43]. Additionally some studies suggest that the gut microbiota can contribute to obesity by inducing a reduction in fat oxidation and an increase in fat storage [43], associated with a relative reduction in the expression of PGC1 alpha and in AMPK phosphorylation. This mechanism is less probable in our animal model, because the RQ of TLR2 KO mice was identical to that of control mice, showing that they were oxidizing fat in the same proportion of controls, and also the tissue levels of PGC1alpha and also the phosphorylation of AMPK were similar in liver and muscle of controls and TLR2 KO mice.

The article "Gut Microbiota Is a Key Modulator of Insulin Resistance in TLR 2 Knockout Mice" was retracted in 2016. Reasons: errors in the images; duplicated images.

Another possible mechanism that could induce insulin resistance in obesity is the increased level of LPS, which is observed in HFD mice [11],[44]. Notably, although TLR2 KO mice were fed on standard rodent chow, they presented higher circulating levels of LPS. Since the microbiota of these mice had a predominance of Firmicutes, which are gram-positive, and do not have LPS in the outer membrane, the increase of LPS circulating levels is certainly not the consequence of a microbiota that produces more LPS. However, the microbiota observed in obesity and also in TLR2 KO mice may increase gut permeability and LPS absorption [45]–[47]. Importantly, as observed in obese animals, which present a significant reduction in Bifidobacteria [48],[49], in the microbiota of lean TLR2 KO mice this genera was reduced compared with the controls. In this regard, the supplementation of Bifidobacteria has been linked to an improvement in the gut barrier function and to reduced levels of LPS [31],[50],[51]. In order to prove that the increased circulating LPS levels of TLR2 KO mice were related to gut permeability, we administered LPS orally to these mice and observed that, in addition to higher basal LPS levels, these animals also showed a higher peak of LPS 1 h after oral gavage of this lipopolysaccharide.

Previous data showed that TLR2 regulates tight junction (TJ)-associated intestinal epithelial barrier integrity and that TLR2 deficiency predisposes to alterations of TJ-modulated barrier function leading to perpetuation of mucosal inflammation [52],[53]. In this regard, our data also demonstrated that, in TLR2 KO mice, there is a reduction in ZO-1 in the small intestine and in the colon, reinforcing that there are alterations in epithelial integrity and gut permeability in these mice. Taken together, these results suggest that the interactions between the predisposition of TLR2 KO mice to alterations in barrier function and the microbiota may have an important role in the increased circulating LPS levels observed in these mice.

The article "Gut Microbiota Is a Key Modulator of Insulin Resistance in TLR 2 Knockout Mice" was retracted in 2016. Reasons: errors in the images; duplicated images.

In accordance with alterations in gut permeability, Kellermayer et al. recently investigated the epigenomic and metagenomic consequences of *Tlr2* deficiency in the colonic mucosa of mice in order to understand the biological pathways that shape the interface between the gut microbiota and the mammalian host. The results showed epigenomic and transcriptomic modifications associated with alterations in mucosal microbial composition and the abundance of many bacterial species were found to differ between WT and TLR2 KO animals. The expression of genes involved in the immune system was modified in the colonic mucosa of TLR2 KO mice, which correlated with DNA methylation changes. This pioneer study demonstrates that significant microbiota shifts associate with epithelial epigenetic changes influenced by the host genome [54].

In order to confirm that gut microbiota was inducing insulin resistance in TLR2 KO mice, we treated these mice with antibiotics for 15 d and showed that this treatment dramatically reduced the gut microbiota and also changed its composition. In parallel, there was an improvement in insulin action, characterized by an increased glucose infusion rate during the glucose clamp, and also an improvement in insulin signaling in the liver, muscle, and adipose tissue. In the TLR2 KO mice treated with antibiotics, we also observed a marked reduction in LPS levels. When we performed gut microbiota transplantation of TLR2 KO mice to *Bacillus*-associated WT mice, which are colonized only by the genus *Bacillus* and are capable of receiving a different microbiota from other mice, the complex composition of the transferred organism was preserved. The transplanted TLR2 KO mice microbiota conferred more weight gain, glucose intolerance, and reduced insulin sensitivity and signaling, associated with increased LPS circulating levels. These data reinforce the hypothesis that the TLR2 KO mice microbiota are able to induce changes in the gut permeability, in turn increasing serum LPS levels, associated with insulin resistance.

The increase in LPS may induce insulin resistance by counteracting insulin signaling, as previously demonstrated [11],[55],[56]. However, the insulin resistance observed in TLR2 KO mice has unique characteristics. There was activation of TLR4 in the liver, muscle, and adipose tissue, associated with ER stress and JNK activation, but no activation of the IKKβ-IκB-NFκB pathway. It was previously described that there is cooperation between TLR4 and TLR2 signaling. This cooperation is evident when LPS is injected in TLR2 KO mice. After the first bolus of LPS, TLR2 KO mice show a robust signal for genes encoding innate immune proteins in the brain. However, the second LPS infusion failed to trigger TNFalpha in TLR2 KO mice. These results indicate that TLR2 is involved in the second wave of TNFalpha expression after LPS and that there is an elegant cooperation between TLR2 and TLR4 [57]. Our results extended these data by showing that the chronic elevation in LPS levels in TLR2 KO mice was not able to increase IKK/IkB/NF-kB pathway and TNFalpha and IL-6 production, but induced an increase in JNK activation in liver, muscle, and adipose tissue of these mice. These data suggest that chronic activation of TLR4 by low doses of LPS is sufficient to increase JNK activation, but the activation of IKK/IkB/NF-kB pathway may also depend on the cooperation between TLR2 and TLR4.

The article "Gut Microbiota Is a Key Modulator of Insulin Resistance in TLR 2 Knockout Mice" was retracted in 2016. Reasons: errors in the images; duplicated images.

The absence of activation of the NFκB pathway and the reduced levels of TNFα and IL-6 make the insulin resistance of TLR2 KO mice different from that observed in DIO mice or in ob/ob mice. We can, thus, suggest that the increase in LPS circulating levels caused activation of TLR4, induced ER stress and JNK activation accompanied by increased IRS-1 serine 307 phosphorylation in the liver, muscle, and adipose tissue, leading to a reduction in insulin sensitivity and signaling and conferring the phenotype observed in the TLR2 KO mice. Phosphorylation of IRS-1 on serine residues interferes with the subsequent insulin-stimulated tyrosine phosphorylation of IRS-1 by IR [58] and IRS-1 can also mediate inhibition of the insulin receptor tyrosine kinase activity [55], and also with downstream signaling as Akt phosphorylation. This insulin signaling pathway is crucial for the metabolic effects of insulin on glucose metabolism [59]. The pharmacological or genetic blockage of TLR4, of ER stress, or of JNK improved action and signaling of insulin in TLR2 KO mice, confirming that this sequence of events has an important role in the insulin resistance of these animals.

Regulatory T cells, a small subset of T lymphocytes, are thought to be one of the body's most important defenses against inappropriate immune responses [60],[61] and can influence the activities of cells of the innate immune system [62]–[64]. Previous data showed that regulatory T cells were highly enriched in the abdominal fat of control mice and reduced at this site in animal models of obesity. This reduction in obesity of regulatory T cells influenced the inflammatory state of adipose tissue and certainly contributes to insulin resistance. Our data showing that in TLR2 KO mice there is a reduction in regulatory T cell in visceral adipose tissue may suggest that this modulation may also contribute to the insulin resistance observed in these animals.

The article "Gut Microbiota Is a Key Modulator of Insulin Resistance in TLR 2 Knockout Mice" was retracted in 2016. Reasons: errors in the images; duplicated images.

The development of obesity and insulin resistance in humans is thought to be promoted by a HFD. Feeding TLR2 KO mice with a HFD for 8 wk caused a marked increase in body weight and in fasting plasma glucose, with levels of over 400 mg/dl at 2 h during the glucose tolerance test, demonstrating that these animals developed not only a more severe form of insulin resistance but also diabetes. The alterations in insulin signaling in tissues also showed a marked down-regulation, in parallel with a higher activation of JNK compared to their controls on HFD. Interestingly, the absence of activation of the IKKβ-IκB-NFκB pathway, described in TLR2 KO mice on standard rodent chow, was also observed when these mice were on HFD. These results demonstrate that the insulin resistance, and later the increase in body weight observed in TLR2 KO mice, is exacerbated by HFD.

A recent report demonstrated that genetically deficient TLR5 mice exhibit hyperphagia, hyperlipidemia, insulin resistance, and increased adiposity [30]. These metabolic alterations correlated with changes in the composition of the gut microbiota. Our model, although showing similar features, presented different aspects that may suggest that different mechanisms may be operating in TLR5 or TLR2 KO mice. First, TLR2 KO mice did not present hyperphagia, and the difference in body weight starts only when these animals are 16 wk old. In the TLR5 KO mice, the insulin resistance is not dependent on TLR4, but in TLR2 KO mice there is an increase in circulating LPS and activation of TLR4. It is possible that these differences not only represent differences in genetic defects but also differences in gut microbiota between these mice.

In conclusion, we may suggest that the loss of TLR2 in conventionalized mice results in a reminiscent phenotype of metabolic syndrome, characterized by a clear difference in the gut microbiota, which induces insulin resistance, subclinical inflammation associated with ER stress, glucose intolerance, and later obesity, which is reproduced in WT by microbiota transplantation and can be reversed using antibiotics. Our results emphasize the role of microbiota in the complex network of molecular and cellular interactions that bridge genotype to phenotype and have potential implications for a wide array of common human disorders involving obesity, diabetes, and even other immunological disorders.

## Materials and Methods

### Materials

Human recombinant insulin was from Eli Lilly (Indianapolis, Indiana, USA). Reagents for SDS-PAGE and immunoblotting were from Bio-Rad. HEPES, phenylmethylsulfonyl fluoride, aprotinin, dithiothreitol, Triton X-100, Tween 20, glycerol, and bovine serum albumin (fraction V) were from Sigma. Protein A-Sepharose 6MB was from GE Healthcare, and nitrocellulose paper (BA85, 0.2 µm) was from Amersham Biosciences. The reagents for the chemiluminescence labeling of proteins in blots were from Amersham Biosciences. Sense and antisense oligonucleotides specific for TLR4 (sense, 5′-C TGA AAA AGC ATT CCC ACC T-3′ and antisense, 5′-A GGT GGG AAT GCT TTT TCA G-3′) were produced by Invitrogen Corp. (Carlsbad, CA). Antibodies against β-actin (mouse monoclonal, sc-8432), TLR4 (rabbit polyclonal, sc-30002), phospho [Ser307]-IRS-1 (rabbit polyclonal, sc-33956), phospho [Tyr941] (goat polyclonal, sc-17199), IRS-1 (rabbit polyclonal, sc-559), phospho [Ser 473]-AKT (rabbit polyclonal, sc-33437), AKT1 (goat polyclonal, sc-1618), phospho [Thr 981]-PERK (rabbit polyclonal, sc-32577), PERK (goat polyclonal, sc-9477), phospho-JNK (mouse monoclonal, sc-6254), JNK1 (mouse monoclonal, sc-1648), phospho[Tyr1162/1163]-Insulin Receptor (rabbit polyclonal, sc-25103), Insulin Receptor β (goat polyclonal, sc-31369), UCP1 (goat polyclonal sc-6529), and MyD88 (goat polyclonal, sc-8197) were from Santa Cruz Biotechnology, Inc. (Santa Cruz, CA). Antibody against ZO-1 was from Abcam (AB96594) (Cambridge, MA). Antibodies against phospho [Thr172]-AMPKα (rabbit polyclonal, #2531), AMPKα (rabbit polyclonal, #2532), and IκB-α (rabbit polyclonal, #9242) were from Cell Signaling Technology (Beverly, Massachusetts, USA).

The article "Gut Microbiota Is a Key Modulator of Insulin Resistance in TLR 2 Knockout Mice" was retracted in 2016. Reasons: errors in the images; duplicated images.

### Mice

TLR2-deficient mice, also called TLR2 knockout (KO) mice, were obtained by Dr. Akira [65] and were kindly provided by Dr. Ricardo Gazzinelli [66] and maintained on a C57BL/6J genetic background. Studies were carried out using male TLR2 KO mice that were age matched with C57BL/6J and obtained from the University of Campinas Breeding Center. C57BL/6J and the TLR2 KO mice have the same origin and have been raised in the same institution (UNICAMP) and in the same room, at University of Campinas Breeding Center. The C57BL/6J strain was generated by backcrossing mice carrying the TLR2 KO mutation 10 times to C57BL/6J inbred mice [67]. TLR2-deficient mice are viable and fertile. The control and the knockout mice used for the experiments were littermates, obtained from a heterozygote × heterozygote cross, from the same mother, from the same cage, in order to have standard conditions for all animals. The investigation was approved by the ethics committee and followed the university guidelines for the use of animals in experimental studies, and experiments conform to the Guide for the Care and Use of Laboratory Animals, published by the U.S. National Institutes of Health (NIH publication no. 85–23 revised 1996). The animals were maintained on 12 h/12 h artificial light-dark cycles and housed in individual cages. Mice were randomly divided into two groups: control, fed on standard rodent chow (3.948 kcal/Kg^−1^), and HFD, fed on a rich-fat chow (5.358 kcal/Kg^−1^) *ad libitum* for 16 wk. The mice were bred under specific pathogen-free conditions at the Central Breeding Center of the University of Campinas.

The article "Gut Microbiota Is a Key Modulator of Insulin Resistance in TLR 2 Knockout Mice" was retracted in 2016. Reasons: errors in the images; duplicated images.

### Serum Analysis

Mice were fasted for 5 h, at which time blood was collected by the retrobulbar intraorbital capillary plexus. Hemolysis-free serum was generated by the centrifugation of blood using serum separator tubes (Becton Dickinson, Franklin Lakes, New Jersey). Serum insulin, cytokines, leptin, and adiponectin were analyzed by ELISA kits purchased from Linco Research Inc (St. Charles, Missouri).

### Determination of NF-κB Activation

NF-κB p50 activation was determined in nuclear extracts from muscle and adipose tissue by ELISA (89858; Pierce Biotechnology), according to the recommendations of the manufacturer.

### LPS Serum Determination

Serum LPS concentration was determined using a kit based on a Limulus amebocyte extract (LAL kit endpoint-QCL1000; Cambrex BioScience, Walkersville, Maryland), where samples were diluted 1/40 to 1/100 and heated for 10 min at 70°C. Internal control of recovery calculation was included in the assessment.

### Glucose Tolerance Test

After 6 h fasting, mice were anesthetized by an i.p. injection of sodium amobarbital (15 mg/kg body weight), and the experiments were initiated after the loss of corneal and pedal reflexes. After collection of an unchallenged sample (time 0), a solution of 20% glucose (2.0 g/kg body weight) was administered into the peritoneal cavity. Blood samples were collected from the tail at 30, 60, 90, and 120 min for determination of glucose and insulin concentrations [68].

### Euglycaemic-Hyperinsulinaemic Clamp

After a 6-h fast, a prime continuous (3.0 mU·kg^−1^·min^−1^) infusion of regular insulin was administered in the groups of mice for 2 h from time 0, to raise plasma insulin and maintain it at a steady-state plateau (90–120 min). A variable glucose infusion (10%) was started 5 min after the beginning of the experiment and was corrected, if necessary, to maintain euglycaemia between 5 and 6.1 mmol/l [69]. Blood samples for determination of plasma glucose were obtained at 5-min intervals throughout the study.

### Oxygen Consumption/Carbon Dioxide Production and Respiratory Exchange Ratio Determination

Oxygen consumption/carbon dioxide production and respiratory exchange ratio (RER) were measured in fed animals through an indirect open circuit calorimeter (Oxymax Deluxe System; Columbus Instruments, Columbus, Ohio), as described previously [70].

The article "Gut Microbiota Is a Key Modulator of Insulin Resistance in TLR 2 Knockout Mice" was retracted in 2016. Reasons: errors in the images; duplicated images.

### Measurement of Food Intake

Standard chow or HFD was given and food intake was determined by measuring the difference between the weight of chow given and the weight of chow at the end of a 24-h period. This procedure was performed during 5 d, with 8-wk-old mice, using metabolic cages for a single mouse (Tecniplast, Italy), obtaining an average of food intake per cage per day. This average was also normalized for body weight.

### 4-Phenyl Butyric Acid (PBA) Treatment

PBA is a chemical chaperone and evidence suggests that it relieves endoplasmic reticulum stress [71]. For acclimation, mice received 100 µl phosphate buffered saline (PBS) twice daily (8 a.m. and 6 p.m.), by gavage, for 3 d. Following the acclimation period, PBA was administered twice daily in two divided doses (500 mg/kg at 8 a.m. and at 6 p.m., total 1 g/kg/day) by gavage for 10 d. Control groups received the same volume of vehicle instead of PBA at the same treatment points [33].

### SP600125 Treatment

SP600125, a potent and selective inhibitor of JNK, was dissolved in a 7% (in PBS) Solutol HS-15 solution and administered intraperitoneally (30 mg/kg/day) for 5 d [72].

### TLR4 Inhibition

In order to inhibit the expression of TLR4, two methods were used: pharmacological inhibition, using 2.4 mg/kg/day ethyl(6R)-6-[N-(2-chloro-4-fluorophenyl)sulfamoyl]cyclohex-1-ene-1-carboxylate (TAK-242) (synthesized at the Chemistry Institute of the University of Campinas) [73], administered daily by gavage during 5 d, and 4 nmol TLR2 antisense oligonucleotide (ASO) inhibition, composed by 5′-AGGTGGGAATGCTTTTTCAG-3′ (sense) and 5′-CTGAAAAAGCATTCCCACCT-3′ (antisense), administered by two daily i.p. injections during 5 d, produced by Invitrogen Corp. (Carlsbad, California, USA).

### LPS Absorption Test

An LPS tolerance test was performed as follows: Fasted mice were gavaged with LPS (300 µg/kg) diluted in water (100 µL) or with water (100 µL). Blood was collected from the cava vein 60 min after gavage. Plasma was separated and frozen [11].

### Intracellular Cytokine Analysis and Foxp3 Staining

The cells were obtained from the adipose tissue and analyzed by flow cytometry. For the determination of the frequency of putative regulatory T cells, the adipose tissue mononuclear cells were stained for the surface marker CD4 (Percp) and after for intracellular transcription factor Foxp3 using APC anti-mouse/rat Foxp3 staining (eBioscience, San Diego, California). The cells were acquired in the FACS Calibur Flow cytometer (BD) and analyzed with FlowJo software.

The article "Gut Microbiota Is a Key Modulator of Insulin Resistance in TLR 2 Knockout Mice" was retracted in 2016. Reasons: errors in the images; duplicated images.

### Antibiotics Treatment

Four-week-old WT and TLR2 KO mice were placed on broad spectrum antibiotics (1.0 g/L ampicillin, 1.0 g/L metronidazole, and 0.5 g/L neomycin) in drinking water for 20 d. During this period mice were monitored for food intake and stool microbiota sequencing.

### Culture-Based Microbial Analysis of Cecal Contents

Total aerobic and anaerobic bacteria were enumerated in selective media and incubation conditions according to Schumann et al. [74]. In brief, cecal samples were diluted in Ringer medium, and total aerobic and anaerobic bacteria were investigated by plating onto nonselective media: TSS medium (Biomerieux, Lyon, France) for 24 to 48 h at 37°C in aerobic and anaerobic conditions. Bacterial numbers were expressed as colony forming units (CFU)/mg cecal content [75].

### Metagenome Profile

Faeces samples were collected in metabolic cages with separated waste collectors, frozen in liquid nitrogen, and kept at −80°C until use. DNA was then extracted using the QIAamp DNA Stool Mini Kit (Qiagen, Hilden, Germany) and quantified. Libraries were synthesized from 500 ng of total DNA following the Rapid Library Preparation Kit (Roche Applied Science, Mannheim, Germany) instructions. These libraries were analyzed in a Bioanalyzer with a High Sensitive DNA Kit (Agilent Technologies Inc., Santa Clara, California, USA), and equimolar pools were made, titrated, and submitted to large volume PCR, following the manufacturer's instructions (Roche Applied Science, Mannheim, Germany). Subsequently, samples were sequenced in GS FLX Titanium, using a GS FLX Titanium PicoTiterPlate Kit combined with a GS FLX Titanium Sequencing Kit XLR70 (Roche Applied Science, Mannheim, Germany). The data obtained from the sequencing were submitted to the MG-RAST server and compared by phylum prevalence among groups [76].

### Microbiota Transplantation

Cecal contents were pooled from 3 TLR2 KO mice and age- and gender-matched WT littermates. Cecal extracts were suspended in PBS (2.5 ml per cecum) and were administered (0.1 ml per mouse) immediately to sterilely packed, 4-wk-old, *Bacillus*-associated, WT mice that were obtained from the Central Breeding Center of the State University of Campinas. Transplanted mice were maintained in sterile cages and monitored for body weight [30].

### Tissue Extraction, Immunoprecipitation, and Immunoblotting

Mice were anesthetized by intraperitoneal injection of sodium thiopental and used 10–15 min later—i.e., as soon as anesthesia was assured by the loss of pedal and corneal reflexes. In some experiments, 3 or 5 min after insulin injection (3.8 units/kg, intraperitoneally), liver or muscle and white adipose tissue were removed, respectively, and homogenized immediately in extraction buffer at 4°C (1% Triton X-100, 100 mm Tris-HCl (pH 7.4), 100 mm sodium pyrophosphate, 100 mm sodium fluoride, 10 mm EDTA, 10 mm sodium orthovanadate, 2.0 mm phenylmethylsulfonyl fluoride, and 0.1 mg of aprotinin/ml) with a Polytron PTA 20 S generator (model PT 10/35; Brinkmann Instruments). Insoluble material was removed by centrifugation for 30 min at 9,000×g in a 70 Ti rotor (Beckman, Fullerton, California) at 4°C. The protein concentrations of the supernatants were determined by the Bradford dye binding method. Aliquots of the resulting supernatants containing 1.0 mg of total protein were used for immunoprecipitation with antibodies against MyD88 overnight at 4°C, followed by SDS-PAGE, transfer to nitrocellulose membranes, and blotting with anti-TLR4. In direct immunoblot experiments, 0.2 mg of protein extracts were separated by SDS-PAGE, transferred to nitrocellulose membranes, and blotted with anti-UCP1, anti-phospho-JNK, anti-IκBα, anti-phospho-PERK, anti-phospho-AKT, anti-phospho [Ser307]-IRS-1, anti-phospho [Tyr941]-IRS-1 (Tyr), anti-phospho-IR, anti-ZO-1, anti-PGC-1α, anti-phospho [Thr171]-AMPK, and anti-IκB-α. The homogeneity of gel loading was always evaluated by blotting the membranes with antibodies against β-actin, IRS-1, AKT, IR, JNK, PERK, and AMPK as appropriate.

The article "Gut Microbiota Is a Key Modulator of Insulin Resistance in TLR 2 Knockout Mice" was retracted in 2016. Reasons: errors in the images; duplicated images.

### Statistical Analysis

Specific protein bands present on the blots were quantified by densitometry. Mean ± S.E. values obtained from densitometric scans and from the other experiments were compared utilizing Student's *t* test for paired samples or by repeat-measure analysis of variance (one-way or two-way analysis of variance) followed by post hoc analysis of significance (Bonferroni test) when appropriate. When analyzing non-linear parameters, we used Mann-Whitney test. A *p*<0.05 was accepted as statistically significant.

## Supporting Information

Figure S1 Taxonomical characterization of WT gut microbiota. Untreated WT stools were analyzed via 16S rRNA analysis.
(TIF)

Figure S2 TLR2 KO mice exhibit taxonomical alterations in gut microbiota. TLR2 knockout (TLR2−/−) mice stools were analyzed via 16S rRNA analysis.
(TIF)

Figure S3 Bacterial phyla distribution in 4-wk-old-WT (A) or –TLR2−/− mice (B). These analyses were obtained by 16S rRNA sequencing.
(TIF)

Figure S4 Bacterial phyla distribution in 16-wk-old-WT (A) or –TLR2−/− mice (B). These analyses were obtained by 16S rRNA sequencing.
(TIF)

Figure S5 Bacterial phyla distribution in 1-y-old-WT (E) or –TLR2−/− mice (F). These analyses were obtained by 16S rRNA sequencing.
(TIF)

Figure S6 Phosphorylation of the insulin receptor in muscle (A), liver (B), and white adipose tissue (WAT) (C). Tyrosine 172 phosphorylation of AMPK in muscle (D), liver (E), and WAT (F). PGC-1α expression in muscle (G), liver (H), and WAT (I). Insulin receptor and AMPK protein expression in muscle, liver, and WAT (lower panels). Equal protein loading in the gel was confirmed by reblotting the membrane with an anti-β-actin antibody (lower panels). Data are presented from six to eight mice per group, from experiments that were repeated at least three times. All evaluations were made with mice on standard chow. * *p*<0.05 between WT mice with or without insulin stimulus; ** *p*<0.05 between WT and TLR2−/− mice with insulin stimulus.
(TIF)

Figure S7 Cecal samples of TLR2 knockout (TLR2−/−) mice were cultured in aerobic and anaerobic environments with or without the treatment with a mixture of antibiotics (AB) (0.5 g/kg neomycin, 1 g/kg metronidazole, and 1.0 g/kg ampicillin). Aerobic bacteria counts went below the detection limit in the groups treated with the AB. TLR2 knockout (TLR2−/−) mice exhibit taxonomical alterations in gut microbiota after the treatment with a mixture of AB (C), compared with controls, without antibiotics treatment (B). Mice stools were analyzed via 16S rRNA analysis. Data are presented from six to eight mice per group, from experiments that were repeated at least three times. All evaluations were made with mice on standard chow. * *p*<0.05 between aerobic bacteria of TLR2−/− mice with or without AB treatment; ** *p*<0.05 between anaerobic bacteria of TLR2−/− mice with or without AB treatment.
(TIF)

Figure S8 Taxonomical characterization of WT gut microbiota after the treatment with a mixture of antibiotics (AB) (0.5 g/kg neomycin, 1 g/kg metronidazole, and 1.0 g/kg ampicillin). WT+AB stools were analyzed via 16S rRNA analysis.
(TIF)

Figure S9 Taxonomical characterization of TLR2−/− gut microbiota after the treatment with a mixture of antibiotics (AB) (0.5 g/kg neomycin, 1 g/kg metronidazole, and 1.0 g/kg ampicillin). TLR2−/− + AB stools were analyzed via 16S rRNA analysis.
(TIF)

Figure S10 Taxonomical alteration obtained from the treatment with antibiotics individually (0.5 g/kg neomycin, 1 g/kg metronidazole, and 1.0 g/kg ampicillin). TLR2−/− mice treated only with metronidazole (A). TLR2−/− mice treated only with neomycin (B). TLR2−/− mice treated only with ampicillin (C).
(TIF)

The article "Gut Microbiota Is a Key Modulator of Insulin Resistance in TLR 2 Knockout Mice" was retracted in 2016. Reasons: errors in the images; duplicated images.

## Abbreviations

ASO: antisense oligonucleotide
CFU: colony forming units
HFD: high-fat diet
IR: insulin receptor
IRS: insulin receptor substrate
KO: knockout
PBA: phenyl butyric acid
PBS: phosphate buffered saline
RER: respiratory exchange ratio
rRNA: ribosomal RNA
T2DM: type 2 diabetes mellitus
TJ: tight junction
TLRs: Toll-like receptors
TLR2: Toll-like Receptor 2
ZO: zonula occludens
